# Analysis of the Effect of the Communication Ability of Nurses in Outpatient Infusion Room on the Treatment Experience of Patients and Their Families

This article has been retracted.

**DOI:** 10.1155/2022/1143662

**Published:** 2022-10-11

**Authors:** Xiuqin Shen, Ying Zhang, Jiao Wei

**Affiliations:** Department of Infusion Center, The First Affiliated Hospital of Soochow University, Suzhou, Jiangsu 215000, China

## Abstract

**Objective:**

To observe the effect of nursing communication ability in outpatient infusion room on the treatment experience of outpatients and their families and analyze whether improving nurses' communication skills can reduce the incidence of doctor-patient disputes.

**Methods:**

According to the results of the communication ability survey, the outpatient nurses in our hospital are divided into groups A (score < 65), B (65 ≤ score < 80), C (80 ≤ score < 95), and D (score ≥ 95). Taking outpatients and their families in our hospital from September 2019 to December 2020 as the research objects, they were divided into corresponding groups according to the nurses who served them. Finally, there were 73 cases in group A, 85 in group B, 92 in group C, and 65 in group D. The mental toughness scale (Connor-Davidson Resilience Scale Chinese (CD-RISC)) scores and Herth Hope Index (HHI) scores of the four groups of patients were compared, and the correlation between nurse communication scores and CD-RISC scores and HHI scores was analyzed. The incidence of negative events (patient-nurse disputes, complaints, etc.) and the results of nursing satisfaction surveys during the visits of the four study groups were also counted.

**Results:**

The four groups of CD-RISC and HHI total scores were ranked from highest to lowest as groups D, C, B, and A, respectively (*P* < 0.05). There was a positive correlation between the resilience dimension scores of the family members' CD-RISC and the toughness, strength, optimism dimension scores of the HHI and the nurses' communication dimension scores (*r* = 0.191-0.472, *P* < 0.05). Besides, the incidence of negative events was higher in group A than in the other three groups, while the satisfaction with care was lower than in the other three groups (*P* < 0.05).

**Conclusion:**

Improving nurses' communication skills in infusion room nursing quality management can improve the mental toughness and hope level of patients' accompanying family members, which is conducive to controlling their emotions and avoiding the occurrence of dispute incidents.

## 1. Introduction

Outpatient infusion rooms are extremely special types of hospital department that does not receive patients with a specific type of disease compared to other departments [1]. Compared to patients in the inpatient department, the length of stay (LOS) of patients in the outpatient infusion rooms is generally shorter, and they are more mobile [2]. The department, however, accommodates a large number of patients and their families, and there are obvious problems such as noisy environment and high crowd density [3]. The survey shows that in tertiary hospitals, the average daily outpatient infusion room receives more than about 300 patients. With the addition of patients' accompanying persons or family members, the average daily population flow in the infusion rooms is basically at 500-800 persons/day [4]. Therefore, the nursing service strategies in the outpatient infusion rooms need to meet both wide applicability and high timeliness that can be completed within a limited working time, which undoubtedly increases the work difficulty of nursing staff in the rooms and brings certain safety risks to nursing safety [5]. Also, the failure to achieve the ideal nursing service work has led to a high incidence of nurse-patient disputes and other incidents [6, 7]. Studies have shown that more than 80% of nurse-patient dispute incidents are caused by miscommunication and mostly occur between patients' families and nurses [8, 9]. We believe that the main cause of disputes between patients' families and nurses is the lack of communication skills of nurses leading to emotional instability of patients' families and sharpening of their relationship. Therefore, improving the communication skills of outpatient nurses may also improve patients' treatment experience and reduce the incidence of adverse events, but there are no studies to test this idea.

To verify our view, we will analyze the correlation between communication skills of nursing nurses and family emotions in infusion rooms, aiming to confirm the importance of nurse communication in outpatient infusion rooms and provide some reference for future nursing strategies.

## 2. Materials and Methods

### 2.1. Nurse Communication Skill Assessment

We assessed the communication skills of nurses in the infusion rooms of our hospital by referring to the Clinical Communication Skills Scale for Nurses by Müller et al. [10]. The scale has 28 assessment items, which was divided into 6 dimensions: building harmonious relationships (6 items), keen listening (5 items), identifying patient problems (5 items), joint participation (4 items), delivering effective information (3 items), and validating feelings (5 items), with scores ranging from frequently to never used on a scale of 1 to 4. A Cronbach's *α* coefficient is 0.84. This time, 30 nurses participated in the survey. Based on the results of nurses' communication scores, they were divided into groups A (score < 65, *n* = 7), B (65 ≤ score < 80, *n* = 9), C (80 ≤ score < 95, *n* = 8), and D (score ≥ 95, *n* = 6).

### 2.2. Research Subjects

A total of 315 family members of patients receiving care in the infusion rooms of our hospital from September 2019 to December 2020 were considered as the study population. The subjects were included in different groups according to different communication skills of the nurses who performed the nursing services, with 73 cases in the group A, 85 in group B, 92 in group C, and 65 in group D.

### 2.3. Inclusion and Exclusion Criteria

Inclusion criteria are as follows: (1) one family member per patient; (2) those were husband and wife, parents, children, and siblings; (3) age: 18-60 years old; and (4) patients and their family members signed an informed consent form. Exclusion criteria are as follows: (1) family members with professional nursing work experience; (2) presence of visual, hearing, speech, and physical dysfunction; and (3) those with a history of mental illness.

### 2.4. Methods

The Chinese version of the Connor-Davidson Resilience Scale Chinese (CD-RISC) and the Herth Hope Index (HHI) scale was used in this research. At the same time, this study implemented an accountable care method. It divides nurses' areas of responsibility, so that they could serve the patients and their families in a certain area on a fixed basis, ensuring that one nurse would perform nursing interventions throughout patients' infusion period, and issuing nurses with the Nurse Clinical Communication Skills Scale to assess their communication skills.

### 2.5. Outcome Measures

(1) Mental toughness: the CD-RISC assessment was used, a scale originally developed by Connor and Davidson and finally obtained the version cited in this study after it was introduced, translated, and revised by our scholars according to our national context [11]. A total of 25 items were assessed on the scale, and the dimensions were fixed in 3 areas, resilience (13 items), strength (8 items), and optimism (4 items), and a score of 0 to 4 was assigned according to the never-to-be-so option under each item. This scale is suitable for assessing people who feel stress, frustration, and other psychological states, and patients in this study fit the characteristics of such people and suit this scale, and the Cronbach's *α* coefficient was 0.879. (2) Hope level: the HHI assessment was used, which was originally developed by Herth and was introduced and translated by our scholars to form the HHI scale introduced in this study [12]. There were 12 items on the scale, and the dimensions were temporality and future (T), positive readiness and expectancy (P), and interconnectedness (I) (3 items each), with a scale ranging from 1 to 4 on a scale of strongly disagree to strongly agree. The Cronbach's *α* coefficient was 0.842. Higher scores on both scales were associated with higher levels of psychological resilience and hope in patients' families, demonstrating better emotional stability. (3) Incidence of negative events: the negative events that occurred during the study period were counted, including the number of complaints to the hospital by patients and their families, the number of nurse-patient disputes, and patients leaving the hospital without completing the infusion as required. The incidence of negative events was calculated = number of negative events/total number × 100%. (4) Nursing satisfaction: after patients' infusion was completed, the patients and their families were invited to fill out a nursing satisfaction questionnaire [13], and the results were divided into three options, very satisfied, generally satisfied, and dissatisfied, and total nursing satisfaction was calculated. Total satisfaction = (very satisfied + generally satisfied)/total × 100%.

### 2.6. Statistical Analysis

Data were entered into SPSS 22.0 for statistical analysis, and the attribute data were expressed as (*n* (%)) with *χ*^2^ test. The variable data were expressed as ($\bar{x}\pm s$), and analysis of variance (ANOVA) with least significant difference (LSD) intragroup test was used for comparison between multiple groups. *P* < 0.05 indicates that the difference is statistically remarkable.

## 3. Results

### 3.1. Comparison of General Data of Study Subjects

To ensure the credibility of the experimental results, we first compared the age, gender, and relationship with patients among the four study groups. It revealed that the age, gender, and relationship with patients were seen to be statistically different among the four groups (*P* > 0.05, Table 1), confirming the comparability among the four groups.

### 3.2. Comparison of CD-RISC Scores

Before infusion, the total CD-RISC scores of the families of the four groups of patients were 69.58 ± 10.28, 68.82 ± 12.14, 70.05 ± 11.46, and 69.15 ± 11.33, respectively, with no statistically remarkable differences (*P* > 0.05). After infusion, the total CD-RISC scores of the four groups were ranked from highest to lowest as groups D, C, B, and A, respectively (*P* < 0.05). Among them, the toughness dimension scores were ranked from highest to lowest as groups D, C, B, and A, respectively (*P* < 0.05). The differences in strength and optimism dimension scores between the four groups were not remarkable (*P* > 0.05, Table 2).

### 3.3. Comparison of HHI Scores

The total HHI scores of family members of patients in the four groups before infusion were 20.69 ± 9.15, 21.08 ± 9.33, 20.54 ± 8.92, and 21.17 ± 8.61, respectively, with no statistically marked difference (*P* > 0.05). The four groups were ranked from highest to lowest in terms of HHI dimension scores and total scores as groups D, C, B, and A (*P* < 0.05, Table 3).

### 3.4. Correlation of CD-RISC and HHI Scores with Nurses' Communication Skill Scores

There was a positive correlation between the resilience dimension scores of patient family members' CD-RISC and the T, P, and I dimension scores of the HHI and the nurses' communication dimension scores (*r* = 0.191-0.472, *P* < 0.05). Scores on the strength and optimism dimensions of patient families' CD-RISC were positively correlated with scores on the establishment of rapport, keen listening, and identification of patient problem dimensions of the nurse communication scores (*r* = 0.189-0.249, *P* < 0.05), but not with the coparticipation, effective delivery of information and validation of feeling dimensions of the nurse communication scores (*P* > 0.05, Table 4).

### 3.5. Incidence of Negative Events

According to statistics, it can be seen that there is no significant difference in the incidence of adverse events between groups B, C, and D (*P* > 0.05), while the incidence in group A was higher than the other three groups (*P* < 0.05, Table 5). Among them, group D did not have any negative events, while both groups B and C had complaints, but no nurse-patient disputes or patients leaving the hospital without completing the infusion. In contrast, there were two cases of nurse-patient disputes in group A patients, while complaints and patients leaving the hospital before completing the infusion also occurred.

### 3.6. Comparison of Nursing Satisfaction Survey Results

The nursing satisfaction survey manifested that the total nursing satisfaction of the study subjects in group D reached 95.38%, which was the highest among the four groups (*P* < 0.05), while no difference in nursing satisfaction was seen between groups B and C (*P* > 0.05). The nursing satisfaction of group A was lower than that of group B and group C (*P* < 0.05, Table 6).

## 4. Discussion

Intravenous infusion generally needs to be maintained for more than half an hour, and the infusion time is longer for individual drugs with greater endothelial irritation and adverse effects on gastrointestinal and cardiac organ functions, etc. Long-term restricted mobility will increase the agitation of patients and accompanying family members. At the same time, the number of patients receiving intravenous infusion in the infusion rooms is high, but the number of nurses is limited. The pressure of busy work makes it difficult for nurses to take care of all aspects of patients' needs, which causes dissatisfaction among their families and induces nurse-patient disputes [14–16]. At present, in order to reduce adverse events in infusion rooms, researchers have proposed many methods, such as changing the management system of the infusion rooms and increasing the number of nurses in infusion rooms [17–19]. But they have not achieved better results. Therefore, this study explored the relationship between nurses' communication ability and family satisfaction, which not only confirmed the importance of nurses' communication ability in infusion room nursing for the first time but also provided a reference for designing a new infusion room nursing model.

The CD-RISC and resilience dimension scores of the four groups in descending order were groups D, C, B, and A. It was seen that after receiving good communication, the families had better mental resilience while accompanying the patients waiting for the infusion to be completed. But the differences in the scores of strength and optimism dimensions in the four groups of mental toughness assessment were small (*P* > 0.05). Combined with the content of the CD-RISC scale, the reasons for this are as follows: (1) the strength dimensions, such as “I feel empowered by coping with stress” and “I have worked hard to achieve my goals,” assessed the psychological attributes of the families and were not influenced by nurse-patient communication, so the strength dimensions did not show differences between groups. (2) The optimism dimension of “Sometimes fate or God can help” is the strength of one's own beliefs, and “I can see the humorous side of things” is related to personal experiences and coping styles, and a short period of nursing communication in the infusion rooms does not affect the assessment results of these items. (3) In the resilience dimension, the nurse's good communication skills could provide the patient's family with a channel to “seek help,” strengthen the belief in “achieving goals,” and speed up the processing of “unhappy emotions,” which had a greater impact on the family's score in this dimension and had a greater impact on the final mental toughness level.

The total HHI score and each dimension score of the four groups were ranked from highest to lowest as groups D, C, B, and A. It is evident that nurses' communication skills can improve the positive coping emotions of patients' families. The main reason analyzed by the researchers was that effective communication between nurses and patients deepened the knowledge of the families about patients' condition and nurses' work, so that they had a clearer perception of the whole process of their loved ones' illness and infusion and had a clear direction and confidence in the psychological coping process [20].

Also, in the correlation analysis for nurses' nursing and patients' CD-RISC and HHI scores, it was learned that there was a positive correlation between the total CD-RISC score and resilience dimension scores of families, and the total HHI score and scores of each dimension and nurses' communication scores of each dimension, which was consistent with the above discussion. But ratings on the strength and optimism dimensions of the families' CD-RISC were positively correlated with ratings on the establishing rapport, listening acutely, and identifying patient problems dimensions of the nurses' communication skills. It was inferred that although the overall effect of nurse-patient communication on the strength and optimism dimensions of the families' CD-RISC was negligible, maintaining a harmonious relationship with them, listening carefully to their questions, and answering them well could still contribute positively to their optimistic way of thinking to some extent.

Observing the incidence of negative events in each study group, we found that group A had the highest incidence of negative events, which also suggested that the communication of our infusion room care largely determined the incidence of negative events. Although no difference was seen in the incidence of negative events among the three groups B, C, and D, it was still evident that there was no case of negative events in group D. This demonstrates the importance of maintaining effective, high-quality communication to improve the quality of nursing. In a previous study, we also found that good communication can enhance patients' and families' trust and dependence on health care professionals [21], which can also corroborate our view. Through the nursing satisfaction survey, we also found that the subjects in group D gave the highest satisfaction rating, which again shows that nursing with better communication skills can gain higher recognition from patients and their families. This is a good indication of the extreme importance of improving nurses' communication skills in outpatient infusion rooms in the future.

Nevertheless, because no randomized controlled trial was conducted, the idea that nurse communication skills can definitively enhance the treatment experience of patients and their families in infusion rooms needs to be further substantiated. What is more, it was mentioned in a previous study that the incidence of nurse-patient disputes is related to the quality of service provided by nursing staff on the one hand and the literacy of patients and their families on the other [22]. Thus, we also needed to capture the educational level of the subjects included in the study and further break it down to determine the role of nurses' communication skills in it. Finally, there are no unified nursing guidelines for infusion rooms in clinical practice, and there may be more areas for improvement and refinement in the process of improving the quality of nursing in infusion rooms, which will also be the focus of our subsequent research.

## 5. Conclusion

Improving nurses' communication skills in the quality management of infusion room care can improve the mental toughness and hope level of patients' accompanying family members and control their emotions in a smoother situation, which is conducive to reducing the incidence of nurse-patient disputes.

## Figures and Tables

**Table 1:** General data of patients' families in the four groups ($\bar{x}\pm s$, *n* (%)).

Groups	Cases	Gender		Age (year)	Relationships with patients			
		Male	Female		Couples	Parents	Children	Brothers/sisters
Group A	73	25 (34.25)	48 (65.75)	46.81 ± 18.29	31 (42.47)	20 (27.40)	17 (23.29)	5 (6.85)
Group B	85	31 (36.47)	54 (63.53)	47.59 ± 15.24	38 (44.71)	23 (27.06)	18 (21.18)	6 (7.06)
Group C	92	39 (42.39)	53 (57.61)	45.91 ± 17.41	41 (44.57)	25 (27.17)	20 (21.74)	6 (6.52)
Group D	65	18 (27.69)	46 (70.77)	46.28 ± 16.95	29 (44.62)	16 (24.62)	15 (23.08)	5 (7.69)
*F*/*χ*^2^		3.687		0.158	0.378			
*P*		0.297		0.925	>0.999			

**Table 2:** Comparison of CD-RISC scores of family members of patients in the four groups ($\bar{x}\pm s$, score).

Groups	Cases	Toughness	Strength	Optimism	Total scores
Group A	73	36.71 ± 5.95	29.14 ± 6.58	12.42 ± 3.05	78.27 ± 7.49
Group B	85	38.63 ± 5.22	29.37 ± 6.11	12.66 ± 3.11	80.66 ± 7.63
Group C	92	40.28 ± 5.17	30.71 ± 7.20	13.02 ± 3.62	84.01 ± 7.85
Group D	65	42.08 ± 5.95	31.12 ± 7.14	13.36 ± 3.28	86.56 ± 5.09
*t* value/*P* value_(A-B)_		-2.161/0.032	-0.288/0.820	-0.488/0.626	-1.980/0.049
*t* value/*P* value_(A-C)_		-4.120/<0.001	-1.445/0.150	-1.132/0.259	-4.760/<0.001
*t* value/*P* value_(A-D)_		-5.292/<0.001	-1.695/0.092	-1.744/0.083	-7.510/<0.001
*t* value/*P* value_(B-C)_		-2.112/0.036	-1.330/0.185	-0.707/0.481	-2.875/0.005
*t* value/*P* value_(B-D)_		-3.774/<0.001	-1.615/0.108	-1.334/0.184	-5.383/<0.001
*t* value/*P* value_(C-D)_		-2.018/0.045	-0.353/0.725	-0.602/0.548	-2.299/0.023

**Table 3:** Comparison of HHI scores of family members of patients in the four groups ($\bar{x}\pm s$, score).

Groups	Cases	Temporality and future	Positive readiness and expectancy	Interconnectedness	Scores
Group A	73	9.82 ± 2.37	8.54 ± 2.36	9.20 ± 2.55	27.56 ± 7.61
Group B	85	10.62 ± 2.64	9.33 ± 2.60	10.04 ± 2.73	29.99 ± 7.74
Group C	92	11.40 ± 2.43	10.14 ± 2.81	10.87 ± 2.82	32.41 ± 8.35
Group D	65	12.18 ± 2.39	11.03 ± 2.72	11.79 ± 2.90	35.00 ± 7.61
*t* value/*P* value_(A-B)_		-1.990/0.048	-1.987/0.049	-1.988/0.049	-1.983/0.049
*t* value/*Pvalue*_(A-C)_		-4.194/<0.001	-3.895/<0.001	-3.940/<0.001	-3.853/<0.001
*t* value/*P* value_(A-D)_		-5.816/<0.001	-5.758/<0.001	-5.583/<0.001	-5.733/<0.001
*t* value/*P* value_(B-C)_		-2.047/0.042	-1.986/0.049	-1.987/0.048	-1.995/0.048
*t* value/*P* value _(B-D)_		-3.735/<0.001	-3.890/<0.001	-3.787/<0.001	-3.957/<0.001
*t* value/*P* value_(C-D)_		-1.995/0.048	-1.981/0.049	-1.990/0.048	-1.985/0.049

**Table 4:** Correlation between patient family members' CD-RISC and HHI scores and nurse communication skill scores (*r*).

	Building harmonious relationships	Keen listening	Identifying patient problems	Joint participation	Delivering effective information	Validation of feelings
Toughness	0.199^∗^	0.410^∗^	0.395^∗^	0.254^∗^	0.400^∗^	0.362^∗^
Strength	0.201^∗^	0.189^∗^	0.197^∗^	0.112	0.110	0.129
Optimism	0.199^∗^	0.223^∗^	0.249^∗^	0.096	0.099	0.117
T	0.316^∗^	0.276^∗^	0.215^∗^	0.259^∗^	0.393^∗^	0.196^∗^
P	0.229^∗^	0.472^∗^	0.360^∗^	0.217^∗^	0.219^∗^	0.262^∗^
I	0.254^∗^	0.359^∗^	0.302^∗^	0.287^∗^	0.191^∗^	0.402^∗^

Note: ^∗^*P* < 0.05.

**Table 5:** Incidence of negative events.

	Nurse-patient disputes	Complaints	Patient leaves hospital before completing infusion	Total incidence (%)
Group A	2 (2.74)	4 (5.48)	1 (1.37)	7 (9.59)
Group B	0 (0.00)	3 (3.53)	0 (0.00)	3 (3.53)
Group C	0 (0.00)	2 (2.17)	0 (0.00)	2 (2.17)
Group D	0 (0.00)	0 (0.00)	0 (0.00)	0 (0.00)
*χ* ^2^				9.918
*P*				0.019

**Table 6:** Nursing satisfaction survey results.

	Very satisfied	Generally satisfied	Dissatisfied	Total satisfaction (%)
Group A	8 (10.96)	45 (61.64)	20 (27.40)	53 (72.60)
Group B	19 (22.35)	57 (67.06)	9 (10.59)	76 (89.41)
Group C	21 (22.84)	62 (67.39)	9 (9.78)	83 (90.23)
Group D	36 (55.38)	26 (40.00)	3 (4.62)	62 (95.38)
*χ* ^2^				18.680
*P*				0.003

## Data Availability

The data used in the article is obtained from the corresponding author upon reasonable request.
